# Metabolic and Endocrine Changes Determined in Saliva of Adolescents Engaged in Computer Gaming

**DOI:** 10.1155/2020/1649759

**Published:** 2020-12-17

**Authors:** Leonid Vladimirovich Podrigalo, Sergii Sidorovich Iermakov, Wladyslaw Jagiello

**Affiliations:** ^1^Department of Medical Science, Kharkov State Academy of Physical Culture, Kharkov, Ukraine; ^2^Department of Sport, Gdansk University of Physical Education and Sport, Gdansk, Poland

## Abstract

Passion for computer games negatively affects the health level of schoolchildren. Among the approaches to monitoring the functional state of such schoolchildren, the most informative and painless is the study of the saliva. The study involved 45 children, aged 14.00 ± 0.21 years, and divided according to the contact's intensity with computer games. The following indicators of lipid peroxidation (LPO) were determined in the saliva: indicators of the antioxidant (AO) system, concentration of immunoglobulin A, and hormonal indicators. The significant increases in the catecholamine (adrenaline) level for 2.3 times and biogenic amine–serotonin for 35.5% and increase in the LPO-DC product concentration in gamers for 75.8% were revealed. The study of the schoolchildren's homeostasis peculiarities confirmed the adequacy of the use of biochemical techniques to assess the condition of children gamers. They have a prenosological condition. This is reflected in the increase in LPO intensity, failure of the protective AO system, imbalance of hormonal state, and immunity deterioration. Information on the evaluation of the LPO activity processes and the AO system condition and the degree of the balance's shift between prooxidants and antioxidants in biological substrates can be considered objective and very sensitive indicators of the general condition, activity, and improvement of the regulation and maintenance of homeostasis.

## 1. Introduction

The widespread use of multimedia technologies leads to the intensification of technological progress and significantly affects the population's health. The availability and use of mobile phones, game consoles, DVD players, television, computers, and tablets have risen exponentially over the past few decades.

Even a brief listing of the basic facts about computer games testifies to the rapid development of this industry. So, in 1958, the first game, a tennis simulator, was created at the Brookhaven National Laboratory. In 1961, MTI (Massachusetts Institute of Technology) created the first computer game Space Wars, a combat simulator. The first arcade game Colossal Cave Adventure was created in 1971. In 1977, Atari launched the first video game consoles. In 1995, the first online chat on the World Wide Web was created, and in 2002, their sales reached $10 billion [1, 2].

Fomby et al. [3] emphasize that mobile digital devices with an Internet connection have changed the use of technology by teenagers in the United States over the past decade. There is a lack of information on the impact of these changes on various health-related behaviors. It also confirmed the increase in time spent on contacts with multimedia technologies. This leads to a decrease in a teenagers' physical activity.

Marouf et al. [4] report that media use by children has particularly increased. The study showed a significant correlation between having a TV in the child's room and the number of sleep hours per day, between the child's physical activity and the smart gadgets' using.

The physical and psychological consequences of computer games cannot be ignored. The duration of the game is correlated with increased aggression, decreased mental health, and a higher body mass index. The results of an online survey conducted by Alshehri and Mohamed [5] confirmed the negative correlation between games and men's health and physical activity. It is concluded that it is necessary to make a profound study of the games' influence on the different segments of society. A similar conclusion was made in a study by Breuer et al. [6].

A study by Kiselev reports on the deterioration of visual-spatial abilities in children due to addiction to computer games [7].

The high prevalence of Internet-related disorders has necessitated their inclusion as new diagnoses in the International Classification of Diseases ICD-11. Internet-related disorders have been clinically described as excessive and poorly controlled online behaviors that are causing detrimental consequences and result in decreasing psychosocial functioning. Müller et al. [8] determine that one of the leading places among such disorders goes to computer games.

Choi et al. [9] studied the possibility of Internet addiction development in schoolchildren. The addiction development was observed with an increase in contacts with multimedia. People with a high risk of addiction had more pronounced negative trends in intellectual and motor indicators.

Another recent study reports the dangers of excessive contact with computer games. The authors identify the main risk factors for health—the development of addiction, increased contact time, and an unhealthy environment [10].

The results of the research by Osipov et al. [11] emphasize the importance of computer technology in the education and leisure of youth, the necessity to regulate contacts with multimedia technologies.

The other research [12] confirmed the correlation between physical activity of varied intensity, computer and video games, and TV watching in Brazilian teenagers. A similar study was conducted by Koçak [13]. The existence of an inverse correlation between Internet addiction and regular physical activity in students was confirmed, and the possibility of using regular physical activity as a preventive and health-improving means of Internet addiction was concluded. The results obtained by Kudryavtsev and Kramida [14] confirm the correctness of such assumption. Qigong training help reduce computer addiction.

The condition monitoring of certain categories of person demands the selection of specific and informative criteria. Kalina and Jagiełło [15] emphasized the need for an integrated innovative approach in the health-related indicators' selection. The methodologies used to determine indicators should be simple, reliable, and meet the methodological criteria.

Subjective methods based on self-assessment are most often used in assessing the impact of multimedia technologies on health. Thus, Daĝal and Bayindir [16] offered to assess the impact of computer games on the children's condition using a special scale.

Almost one criterion is used to include users to the group of active players. It is the frequency and duration of games, assessed by the results of the survey. Song et al. [17] assessed the teenagers' lifestyle by the questionnaires. The games' playing for 1 day a week was a criterion for inclusion in the group of active players. It is concluded that 40% of high school pupils in the United States are active players (gamers). They are characterized by a sedentary lifestyle, excess body weight, or obesity compared to inactive players.

In research conducted by Valencia-Peris et al. [18] was assessed the prevalence of computer games in teenagers. The authors assessed differences in lifestyle depending on the intensity degree of this factor. The group of active players includes those who played at least 10 minutes a day. The specific gravity of such teenagers was 25.9%.

In our opinion, the criteria we used to classify children as active players allow us to more effectively assess the impact of this type of activity on health. Bashir and Zara [19] obtained similar data. The authors assessed the correlation between myopia development and the factors influencing it. The most intensive were computer games, TV watching, and reading. The percentage of children playing games or using a computer for 1 hour was 60.72%, 35.66% for 2-4 hours, and 3.62% for >4 hours.

Popow et al. [20] determined that computer game disorders are new and common conditions in modern children and teenagers. The lack of necessary diagnostic tools and developed preventive strategies was emphasized. In this regard, the use of the battery of biochemical tests is an informative and objective way of health monitoring.

Some research [21] reported the higher informativeness of biochemical indicators in comparison with physiological. Soyal and Çelik [22] recommended controlling the metabolic changes in the body as an indicator of monitoring of youths' conditions during strength training.

The used battery of tests allows estimating the various metabolic indicators and health conditions from various points of view. A similar battery of tests was used in the research of Volodchenko et al. [23]. The authors studied the condition of the LPO-AOS system and the metabolism peculiarities in the dynamics of martial arts athletes' training.

Computer games can be characterized by other criteria that affect the level of health of young people.

Thus, Gao et al. determined the metabolic equivalents (METs) of several activities typically performed by Chinese youth [24]. A MET value is 3.1 in jumping rope at low effort. The MET value for computer games was ranging from 0.8 to 1.2.

Other authors examined whether screen time (television viewing, video games, and computer games) is associated with cardiometabolic disease (CMD) risk factors in young adults [25]. The findings show that screen time may contribute to the risk of obesity and CMD in young adults.

Wendt et al. performed genetic correlation, Mendelian randomization, and latent causal variable analyses to identify shared genetic mechanisms between psychiatric disorders (Psychiatric Genomics Consortium) and CDU (UK Biobank) [26]. The authors suggest that biological mechanisms underlying CDU contribute to the psychiatric phenotype manifestation.

Voiskounsky [27] emphasizes the importance and relevance of studying the phenomenon of computer games and their influence on the health of a user. The interdisciplinary nature of research and the need to involve different approaches were emphasized.

Thus, the available literature sources confirm the high prevalence of multimedia technologies among schoolchildren and youth. Analysis of the technologies' influence on health must be considered a relevant scientific problem.

Based on the available data, the hypothesis of our study was that excessive contact with computer games leads to disorders of the endocrine system, intensification of oxidative stress, and the gradual formation of a prenosological state.

Based on the above statements, we assumed that increased gaming leads to hormonal and metabolic changes.

The aim of the study is to prove in a controlled study that the metabolic, antioxidant, lipid peroxidation, hormonal, and sIgA changes are related to increased gaming.

## 2. Materials and Methods

### 2.1. Ethics Statement and Participants

This study was approved by the Bioethics Committee for Clinical Research and conducted according to the Declaration of Helsinki (protocol of the Commission on Bioethics of the Kharkov State Academy of Physical Culture No. 32).

The study involved 45 schoolboys, and average age is 14.00 ± 0.21 years.

We informed them about the purpose and test procedures and about the possibility of withdrawal of consent at any time for any reason.

Participants were previously explained about the absence of possible harm to health. Schoolchildren who refused to participate in the work were not involved. The parents of the remaining schoolboys gave written informed consent for their children to participate in the study.

Participants were divided into 2 groups. The selection criterion is the frequency and duration of contacts with computer games, which schoolboys have indicated in the questionnaire. The group of active players consisted of 26 schoolboys. They played at least 5-6 times a week and more than 3 hours a day. The choice of 3 hours as the lower limit for assessing gaming activity is confirmed by research conducted in Ukraine within the framework of the “Health of the Nation 2002-2012” program [28].

The control group consisted of 19 schoolboys who did not play computer games at all. This allowed us to assess the impact of computer games on the biochemical parameters of the saliva. The participants did not have chronic diseases; they belonged to the groups of healthy and practically healthy children according to the data of medical examinations. There were no significant differences in the diet of the participants. The participants denied taking any medications or dietary supplements.

The participants belonged to the group of apparently healthy children according to the results of a dental examination.

### 2.2. The Design of the Study

The work used the generally accepted methods of biochemical analysis [29, 30].

The design of the study involved the determination of 10 biochemical indicators of the saliva. The saliva was collected according to certain rules. All participants rinsed their mouths with distilled water, then collected about 5 mL of saliva in test tubes for 10-15 minutes. No saliva stimulants were used. The samples were placed in a refrigerated thermos and delivered to the laboratory within 2 hours. Then, the samples were centrifuged.

Biochemical tests were performed in a certified laboratory of Kharkiv National Medical University. The determination of diene conjugates (DC) was performed spectrophotometrically. Malonic dialdehyde (MDA) was determined fluorimetrically by reaction with thiobarbituric acid. Catalase activity was determined spectrophotometrically with a substrate of hydrogen peroxide. The concentration of SH groups and reduced glutathione was determined spectrophotometrically with Ellman's reagent. The hormonal link of homeostasis was assessed by the level of adrenaline, serotonin, and thyroid hormones—triiodothyronine and thyroxine. The determination was performed with sets of reagents “AlcorBio” (Russia). Nonspecific resistance was assessed by the concentration of secretory immunoglobulin A (IgA), which was determined by the enzyme-immunosorbent method.

### 2.3. Statistical Analysis

Statistical analysis includes a set of parametric and nonparametric indicators. This allows us to confirm significant differences between the studied groups. The method of correlation matrices allows you to compare groups and to judge the presence of relationships between the studied criteria. The legality of using this method has been confirmed by other studies [23, 31].

Statistical analysis was performed using licensed MS Excel. The following descriptive statistics' indicators were determined: arithmetic means (*M*), standard deviation, and mean error (*m*). The significance of differences between groups was assessed using parametric (Student's *t*-test) and nonparametric (Rosenbaum's criterion *Q*) indicators. The differences were considered significant at *p* < 0.05.

The correlation matrices were constructed, including Pearson coefficients, based on the obtained results. Comparative analysis of correlation matrices was performed using the following indicators: specific gravity of significant and reliable correlations, the labilization/synchronization coefficient (CL), and the average correlation coefficient (ACC). The last two indicators were determined by special formulas given in Zosimov's work [32]:

(1) $$\begin{array}{c} \text{CL}=\left[\frac{n}{N\left(N-1\right)}\right]100\%, \end{array}$$

where *n* is the sum of all significant correlations formed by each indicator of the correlation structure and *N* is the total number of structure's indicators.

(2) $$\begin{array}{c} \text{ACC}=\frac{\sum rj}{n}, \end{array}$$

where *Σrj* is the sum of the values of all significant correlation coefficients of the structure and *n* is the number of significant correlations.

## 3. Results

The obtained results are shown in Table 1.

The results of the control group are shown in column 2; the results of the experimental group are shown in column 3. The results of Table 1 reflect a significant difference in indicators, which is confirmed using parametric Student's *t*-test. We present the values of Student's *t*-test and Rosenbaum's criterion *Q* in the text when they confirm the reliability of the differences between the groups.

The significant differences between the group of active players and children who have no contact with games was determined, in DC (*t* = 8.91, *Q* = 21), catalase activity (*t* = −6.26, *Q* = 20), SH groups concentration (*t* = −2.01, *Q* = 10), reduced glutathione concentrations (*t* = −6.65, *Q* = 23), secretory IgA (*t* = −5.70, *Q* = 10), adrenaline (*t* = 3.15, *Q* = 24), and serotonin (*t* = 2.72). The concentration of DC in the group of active players was 75.8% higher, the catalase activity was 2.23 times lower, the concentration of SH groups was 32% lower, the concentration of reduced glutathione was 73% lower, the secretory IgA level was 40% lower, the adrenaline concentration -2.3 times higher, and serotonin concentration -35.5% higher.

The results of the comparative analysis of correlation matrices are given in Table 2.

The reliable correlations in the group of active players were determined only between the indicators of the antioxidant system: SH groups and reduced glutathione (*r* = 0.51). These parameters had a significant correlation with immunoglobulin A; the value of the coefficient in both cases was *r* = 0.42. The correlation between LPO products and antioxidant system's indicators were weak and unreliable. Significant unreliable correlations were determined between the level of LPO products and the triiodothyronine concentration; the value of the coefficient in both cases was *r* = −0.30. The same nature of the dependency was confirmed between the level of adrenaline and the concentration of immunoglobulin A (*r* = −0.35).

The reliable inverse correlations were determined in the group of no contacts with games between DC and catalase (*r* = −0.57), reduced glutathione (*r* = −0.57), immunoglobulin A (*r* = −0.62), catalase and adrenaline (*r* = −0.51), and adrenaline and immunoglobulin A (*r* = −0.51). The correlation between DC and adrenaline was direct and strong (*r* = 0.72). A similar dependency was determined in DC with serotonin, although less strong (*r* = 0.52).

The analysis of the given data in Table 2 confirms the absence of disorders' prominent features in the studied groups. There is only a tendency to reduce the number of reliable and significant correlations in active players compared to children who do not play computer games. The average correlation coefficient in both groups belonged to the average interval, but in active players, it was lower. The groups of active players are characterized by a decrease in the synchronization/labilization index, which was 5.87 against 9.66 in the control.

The results shown in Figure 1 confirm that prolonged computer games lead to stress and depletion of the protective antioxidant system. This is reflected in a significant (*p* < 0.05) decrease in the concentration of catalase, the level of SH groups, and reduced glutathione.

Child gamers are characterized by a decrease in nonspecific immunity due to a decrease in the concentration of secretory immunoglobulin A (Figure 2).

Prolonged contact with computer games leads to an increase in the concentration of adrenaline in saliva (Figure 2). Figures 1 and 2 reflect a significant difference in the indicators of the studied groups, which is confirmed using parametric Student's test.

The results shown in Figures 1 and 2 confirm that a prenosological state of health is gradually formed in the group of active players. The characteristic manifestations of this condition are imbalance in the LPO-AOS system, gradual depletion and disruption of protective antioxidant mechanisms, a decrease in the level of resistance, and an imbalance of the endocrine system. All these factors significantly reduce the reliability of the body's functioning and increase its vulnerability from adverse factors.

## 4. Discussion

The analysis of the obtained results allows concluding that active players form a prenosological condition as a result of contact with computer games. The reversibility of this condition is confirmed by the absence of significant differences between the final product and LPO-MDA.

The increase in the DC level in active players reflects the increase in LPO intensity due to the increase in intermediates. This determines the stressful character of this type of activity, leading to an increase in the concentration of free radicals in biological fluids, including the saliva.

Increasing the intensity of LPO leads to stress and gradual depletion of the enzymatic link of the antioxidant system. This is reflected by a decrease in the catalase activity, which directly eliminates free radicals. The decrease in the SH group concentration and reduced glutathione shows the decrease in direct and indirect antioxidant actions. In our opinion, it reflects a gradual decrease in the potential of adaptation mechanisms due to constant and long-lasting computer games. Therefore, data to assess the activity of antioxidant defense and LPO and the degree of balance shift in the between prooxidants and antioxidants in biological substrates can be considered objective and very sensitive indicators of the general body condition, activity and regulation system's improvement, and maintenance of homeostasis stable condition.

The integral nature of the body's antioxidant defense predetermines the need to study it under various influences. Akgul and Koz [33] studied the dynamics of antioxidant parameters under conditions of 8-week intense physical activity. The authors confirmed an increase in the activity of the following enzymes: glutathione peroxidase and superoxide dismutase.

The indicators used in our work allow us to assess the integral indicators characterizing human health—the level of oxidative stress, the state of immunity, and the balance of the endocrine system. Comparison of schoolchildren who differ in the frequency and duration of contacts with computer games allows us to assess the severity of health changes.

The importance of antioxidant defense for health disorder prevention was confirmed by Podrigalo et al. [34]. Adequate content of nutrients—antioxidants in the dietary structure—is estimated as an effective factor in healthy recreation.

Constant and prolonged contact with computer games lead to deregulatory changes in children's bodies. This is reflected by a significant (*p* < 0.05) increase in the catecholamine (adrenaline) level and biogenic amine-serotonin in active players. Besides, the increase in serotonin concentration should be assessed as vascular dystonia. This is a prognostically unfavorable sign indicating the formation of prenosological conditions.

The hormonal state determines many factors of homeostasis, such as bone density [35]. The determined changes in hormonal indicators should be assessed as an unfavorable factor from the perspective of the growth and development processes' prediction.

The decrease in the immunoglobulin A concentration in the saliva of active players reflects a decrease in resistance. It is also an unfavorable factor from the perspective of the health condition's prediction. This indicator is an integral criterion of the body's resistance to unfavorable factors. Nazaryan et al. obtained similar results [36]. The authors defined that the functional activity of immunoglobulins depends on not always obvious factors. Their action can lead to a violation of tissue immunity.

Avilova et al. [37] emphasize that one of the factors influencing the activity of the immune system, including the level of immunoglobulins production, is the influence of unfavorable environmental factors. In this context, the environment is contact with multimedia technologies.

The made assumptions are confirmed by the analysis of the determined correlations. The correlations of the antioxidant system reflect their synergism in limiting LPO intensity in active players. The correlation between the immune and antioxidant defense condition indicate their joint activity. The weak and unreliable nature of the correlations between the performance of LPO and the antioxidant system confirms the assumption of stress and depletion of defense mechanisms under the influence of computer stress. The unreliable nature of the correlations among hormone levels, LPO products, and immunoglobulin content was revealed. It does not allow concluding.

However, it can be assumed that there are trends when LPO intensification causes stress on the body's regulatory systems. The expressed game stress causes immune state deterioration.

Analysis of correlations in the group of no contacts with games confirms the done assumptions. Significant inverse correlations between LPO and the antioxidant and immune systems indicate the balance of defense mechanisms in the absence of excessive adverse effects. Direct dependencies of DC with adrenaline and serotonin can be assessed as a synergism of stress factors.

The nature of the identified disorders allows considering them as donosology—an intermediate condition between health and disease. Predictive approaches, including dependence analysis, are widely used in the assessment of such conditions.

Predicting the impact of multimedia technologies on user health is quite common. Buiza-Aguado et al. [38] studied the prevalence of computer game addictions among students. They emphasized the need to develop diagnostic tools and criteria. The use of rating scales allowed to identify people with a high risk of addiction. The multifactor analysis showed that the presence of addiction symptoms was significantly associated with adaptation and psychosocial health deterioration.

Hellstrom et al. [39] assessed the correlation between online gaming and the intensity of depressive, musculoskeletal, and psychosomatic symptoms in adolescents using special questionnaires. It has been found that playing time increasing also raises the probability of these symptoms. It is concluded that excessive playtime contributes to teenagers' health deterioration.

Comparative analysis of correlation matrices allows clarifying and deepening the individual comparison of dependencies between indicators. This method was used by us in assessing the metabolic changes in kickboxing athletes [23] and elite female athletes of synchronized swimming [40]. The obtained results allowed us to assess the adaptive capabilities of athletes and to predict their success level.

In our opinion, these data reflect the peculiarities of the prenosological condition formation in active players as a result of an excessive fascination with computer games. The results of Table 2 support this assumption. The imbalance increase in the system occurs due to a change in the synchronization/labilization indicator, a lower average correlation coefficient, a tendency to a decrease in the specific gravity of significant, and reliable correlations.

The complex of biochemical parameters used allows to adequately assess metabolic changes in the body of children gamers. It can be used to effectively monitor the health status of schoolchildren. The need for such monitoring for this category of the child population was proved in the work of Serduk [28].

The selection of the saliva as the object of examination allows for easy, painless sample collection. This is consistent with the approaches given by Volodchenko et al. [23].

Screening tests and indices are an effective tool for monitoring prenosological conditions [41].

Indices illustrating the state of the LPO-AOS system can be a promising tool for assessing the health of schoolchildren gamers. The validity of this approach was proven in the study by Volodchenko et al. [23].

Prospects for future work should be aimed at substantiating the standards of the indicators used, establishing the relationship between biochemical parameters and the results of functional tests that assess the state of the body's sensory systems.

## 5. Conclusion

Differences in homeostatic indicators were revealed in children belonging to the group of active players in comparison with those who do not have contact with computer games. Activation of the sympathoadrenal system and lipid peroxidation were accompanied by a decrease in antioxidant protection and suppression of nonspecific body resistance. The changes can be interpreted as a violation of regulation and discoordination of adaptive compensatory mechanisms. This allows us to include active players in the risk group, to consider the determined deviations as objective criteria for the prenosological condition development. Further research will be devoted to the development of quantitative criteria for predicting a pronosological state, which is due to the influence of computer games.

Concerning the high prevalence of computer games, the emergence of e-sports, a biochemical study of saliva, may be recommended to assess the players' condition. Further prospect is to develop a scheme for monitoring the health of cyber athletes using biomechanical indicators.

The proved adequacy, informativeness, and accessibility of the saliva use as a subject of study, along with atraumatic, allow to recommend it to implementation as a specific method of health monitoring.

## Figures and Tables

**Figure 1:** Indicators of the enzymatic antioxidant system (EAS) of schoolchildren with different durations of contact with computer games.

**Figure 2:** Indicators of nonspecific immunity (NSI) and hormonal status (HS) of schoolchildren with different durations of contact with computer games.

**Table 1:** Biochemical indicators of schoolchildren's saliva with different frequency of computer game contacts (*M* ± *m*).

Indicator	No contact with games (сontrol group)	Active players (study group)
Malondialdehyde (*μ*mol/L)	3.31 ± 1.54	2.85 ± 0.14
Conjugated dienes (*μ*mol/L)	23.06 ± 1.53	40.55 ± 1.24^∗^
Catalase (*μ*kat/L)	2.28 ± 0.20	1.02 ± 0.05^∗^
SH-groups (mmol/L)	0.74 ± 0.10	0.53 ± 0.02^∗^
Reduced glutathione (mmol/L)	1.09 ± 0.06	0.63 ± 0.03^∗^
Triiodothyronine (nmol/L)	1.65 ± 0.13	1.94 ± 0.24
Thyroxine (nmol/L)	64.24 ± 1.20	59.41 ± 2.44
Secretory IgA (nmol/L)	28.37 ± 1.16	20.26 ± 0.82^∗^
Adrenaline (nmol/L)	1.62 ± 0.14	3.77 ± 0.67^∗^
Serotonin (nmol/L)	190.78 ± 12.94	258.57 ± 21.26^∗^

Note. ^∗^Differences of *t* are significant (*p* < 0.05).

**Table 2:** Indicators of correlation matrices of schoolchildren with different frequency of contacts with computer games.

Group	Specific gravity of significant correlations (%)	Specific gravity reliable correlations (%)	Labilization/synchronization indicator	Average correlation's coefficient
Active players	24.44 ± 6.41	13.33 ± 5.07	5.87	0.33
No contact with games	35.56 ± 7.14	24.44 ± 6.41	9.66	0.43

## Data Availability

The data used to support the findings of this study are available from the corresponding author upon request.
